This article has been retracted.

# A Birth Cohort Study of Neurodevelopmental Outcomes from Birth to 2 Years of Age in Preterm Infants under 34 Weeks of Gestation

**DOI:** 10.1155/2022/7496785

**Published:** 2022-04-13

**Authors:** Hui-Li Li, Ling-Ling Chen, Gang Qian, Wei-Shi Wang, Xiao-Na Feng, Mei-Qiao Yu, Lu-Zhong Ren

**Affiliations:** ^1^Child Health Care Department, Shenzhen Longgang District Maternity and Child Health Care Hospital, Shenzhen 518172, Guangdong, China; ^2^Child Health Care Department, Shenzhen Longgang Central Hospital, Shenzhen 518100, Guangdong, China; ^3^Health Care Department, Shenzhen Longgang District Maternity and Child Health Care Hospital, Shenzhen 518172, Guangdong, China

## Abstract

**Background:**

The tissues and organs of premature infants are immature and easily damaged by external adverse factors, leading to functional development disorders and abnormalities. Besides, the incidence of premature babies in various countries has an increasing trend, with the incidence rate exceeding 10%.

**Objective:**

This study aims to investigate the neurodevelopment and the incidence of various developmental delays, cerebral palsy, autism spectrum disorder, and audio-visual impairment in premature infants under 34 weeks of gestation from birth to 2 years of age, so as to provide the basis for early intervention of premature infants in the clinic.

**Methods:**

A cohort of premature infants was established using 263 premature infants with a gestational age of 28–33 + 6 weeks who were born alive from March 1, 2018, to February 28, 2019, in four tertiary hospitals in Shenzhen. In addition, 263 full-term infants of the same sex who were born in the same period in the four hospitals were randomly selected and paired in a ratio of 1 : 1 as the control group. The subjects were assessed for neurodevelopment using the Gesell test scale at 6, 12, 18, and 24 months after birth (premature infants were corrected for months). We calculated the neurodevelopmental indicators of children in each month of age and the incidence of various developmental delays, cerebral palsy, autism spectrum disorder, and audio-visual impairment in the two groups.

**Results:**

The results of this study showed that the cohort of premature infants with birth gestational age less than 34 weeks had higher adaptive, fine motor, and personal-social energy domain development quotient (DQ) values from the corrected gestational age of 6 months to the corrected gestational age of 24 months after birth compared with the full-term cohort. And it also achieved catch-up growth in neurological development, but the detection rates of neurodevelopmental abnormalities at the corrected gestational age of 12 and 24 months were higher than those in the full-term cohort.

**Conclusion:**

It is important to reduce the disability rate and degree of premature infants by strengthening the systematic management, early promotion and supervision, as well as early intervention for preterm infants with developmental abnormalities who were born at gestational age less than 34 weeks after birth.

## 1. Introduction

In 2012, the World Health Organization (WHO) and other agencies jointly issued the Global Action Report on Premature Delivery, and the report pointed out that the incidence of premature babies in various countries has an increasing trend, with the incidence rate exceeding 10% [1]. With the development of perinatal medicine and the improvement of treatment levels of critical neonates, the survival rate and quality of life of premature infants with extreme survival activity have reached a high level [2]. However, the tissues and organs of premature infants are immature and easily damaged by external adverse factors, leading to functional development disorders and abnormalities. It has been reported in the literature that the smaller the gestational age, the higher the risk of various serious complications, especially nervous system dysfunction, including cerebral palsy and emotional, behavioral, cognitive, and psychological development disorders [3–5], which seriously affect the prognosis. Premature birth misses the critical period of brain development in the last three months of the fetus. This will cause a reduction in the number of nerve cells, and the pathways of dendritic branching, synapse formation, and cortex thickening are interrupted.

In 2016, the General Office of the State Council issued the National Disability Prevention Action Plan. Effective control of birth defects and developmental disability is one of the main actions. Most studies in China and abroad have shown that premature infants with gestational age less than 34 weeks have a high risk of nervous system developmental abnormalities. Therefore, to carry out early neurodevelopment studies on these premature infants is of great significance to explore and promote the neurodevelopment of premature infants and prevent their developmental disabilities.

In this study, a multicenter birth cohort study was conducted on premature infants under 34 weeks of age to explore the neurodevelopment of such premature infants from birth to 2 years of age and the incidence of cerebral palsy, various developmental delays, and visual and auditory impairment, so as to provide a basis for clinicians to carry out early intervention on premature infants and for health administrative departments to make public health decisions on premature infants.

## 2. Objects and Methods

### 2.1. Objects

A cohort of premature infants was established using 263 premature infants with a gestational age of 28–33 + 6 weeks who were born alive from March 1, 2018, to February 28, 2019, in four tertiary hospitals in Shenzhen. Exclusion criteria of research subjects: (1) death within 2 months after birth; (2) suffering from congenital multiple malformations, genetic metabolic diseases, and severe congenital heart disease; and (3) the loss of follow-up within 12 months of gestational age was corrected.

A total of 263 full-term infants of the same sex who were born at the same time in the four hospitals (within one week of the date of birth from the observation group) were randomly selected and paired in a ratio of 1 : 1 as the control group. Inclusion criteria of the control group: (1) gestational age at birth ≥37 weeks and birth weight ≥2500 g and (2) parents were willing to receive health education and could be followed up to 2 years old regularly. Exclusion criteria were the same as those in the premature infant cohort.

### 2.2. Method

#### 2.2.1. Follow-Up Methods and Data Collection

Brainstem auditory evoked potentials and retinopathy of prematurity screening were routinely performed after birth in premature infants. After the premature infant cohort was discharged, the premature infant management specialists from the four hospitals conducted the systematic follow-up in accordance with the “Health Care Work Specifications for Premature Infants” issued by the National Health and Family Planning Commission [6]. Parents under 1 year old were instructed to carry out the intelligent nursing training at the age of 0–1 years according to the recommendation of the Professional Committee for Child Development of China Association of prepotency and child-rearing. They were given the rehabilitation intervention of neurodevelopment therapy in case of motor developmental delay, muscle tension, and posture abnormality during the follow-up of premature infants. The cohort of full-term infants received routine health guidance at the children's health clinics of the four hospitals on a regular basis according to the requirements of the Technical Service Specifications for Children's Health Care issued by the Ministry of Health. The subjects were assessed for neurodevelopment using the Gesell scale at 6, 12, 18, and 24 months after birth (premature infants were corrected for months). The severity of cerebral palsy was assessed at 12 and 24 months of age, respectively. We counted the neurodevelopmental indicators of children in each month of age and the incidence of cerebral palsy, various types of developmental delay, autism spectrum disorder, and visual and auditory impairment in the two groups.

#### 2.2.2. Neurodevelopmental Assessment

*Gesell Development Evaluation*. The evaluation content included five energy regions: gross motor, fine motor, adaptive behavior, language, and personal-social behavior. The observed behavior pattern was identified based on the normal behavior pattern and expressed by age. Then compared with the actual age, the developmental quotient (DQ) was calculated, i.e., DQ = developmental age/actual age ×100, DQ > 85 was classified as normal level, 76–85 as marginal level, and DQ ≤ 75 as developmental delay.

*Diagnosis of Complete Developmental Delay*. With reference to the diagnostic criteria for complete developmental delay in the fifth edition of the Diagnostic and Statistical Manual of Mental Disorders (DSM-5), two or more energy regions DQ ≤ 75 in the Gesell test were required in this study.

*Diagnosis of CP*. The definition, diagnostic criteria, and clinical classification of CP issued by the Drafting Committee of China Guidelines for CP Rehabilitation in 2014 was referred [7].

*Diagnosis of Autism Spectrum Disorder*. The diagnosis of autism spectrum disorder was made by referring to the diagnostic criteria of autism spectrum disorder in the fifth edition of the Diagnostic and Statistical Manual of Mental Disorders (DSM-5) [8].

*Diagnostic Criteria of Retinopathy of Prematurity*: The diagnosis was made by referring to the 2014 edition of Chinese Screening Guideline for Retinopathy of Premature Infants [9].

### 2.3. Statistical Analysis

SPSS23.0 statistical software was used for data processing. The chi-square test was used for intergroup comparison of enumeration data, and the difference was statistically significant with *P* < 0.05. We used mean standard deviation ($\bar{\chi }$ s) to express measurement data, and the one-way analysis of variance was used to compare the mean differences among multiple groups.

## 3. Result

### 3.1. General Run of Things

#### 3.1.1. Enrollment of Premature and Full-Term Infants

A total of 270 premature infants with a gestational age of 28–33 + 6 weeks were born alive in four cooperative units in Shenzhen from March 1, 2018, to February 28, 2019. Among them, seven cases died within two months after birth, with the mortality rate of 2.59%. The effective cases were 263, including 154 males and 109 females. Meanwhile, 263 full-term infants of the same gender were included. To the end of the cohort study, 203 premature infants were followed up in the cohort with the gestational age of (31.3 1.5) weeks and birth weight of (1695.9 414.8) g, 118 males and 85 females, and 60 cases (36 males and 24 females) were lost to follow-up, with the loss of follow-up rate of 22.81% (60/263). 195 full-term infants were followed up in the cohort with the gestational age of (39.0 1.0) weeks. There were 118 males and 81 females with birth weight of (3288.7 407.3) g, and 68 cases (40 males and 28 females) were lost to follow-up, with the loss of follow-up rate of 25.86% (68/263). There was no significant difference in the loss of follow-up rate between the two cohorts (*χ*^2^ = 0.661, *P* = 0.416), and there was no significant difference in the gender ratio between the two cohorts (*χ*^2^ = 0.005, *P* = 0.946).

#### 3.1.2. Completion of the Gesell Test in the Preterm and Full-Term Cohorts

93.10% (189/203) of the preterm cohort and 92.31% (180/195) of the full-term cohort completed the 6-month-old Gesell.

Affected by the novel coronavirus 2020 epidemic, 75.37% (153/203) of the preterm infants in the cohort completed the 12-month corrected gestational age Gesell test, 68.47% (139/203) completed the 18-month corrected gestational age Gesell test, and 84.73% (172/203) completed the 24-month corrected gestational age Gesell test. In the full-term cohort, 84.10% (164/195) of children completed the 12-month Gesell test, 65.64% (128/195) of children completed the 18-month Gesell test, and 80.51% (157/195) of children completed the 24-month Gesell test.

### 3.2. Comparison of Neurodevelopmental Abnormalities at 6, 12, 18, and 24 Months of Age between the Preterm and Full-Term Cohorts

#### 3.2.1. Comparison of Neurodevelopmental Abnormalities at 6 Months of Age between the Two Cohorts

At the corrected gestational age of six months, a cohort of 189 premature infants completed the Gesell test, including 139 cases with normal neurodevelopment and 18 cases with various types of developmental abnormalities, with a detection rate of 9.52% (18/189), including two cases of cerebral palsy (a detection rate of 1.06%, 2/189) and two cases of moderate hearing impairment (a detection rate of 1.06%, 2/189). In 32 cases of developmental limbic state (with two or more energy regions 76 ≤ DQ ≤ 85 margin), the detection rate was 16.93% (32/189).

At the age of six months, a cohort of 180 full-term infants completed the Gesell evaluation, including 141 cases with normal neurodevelopmental status and 24 cases with various developmental abnormalities, with a detection rate of 13.33% (24/180). In 15 cases with neurodevelopmental limbic state, the detection rate was 8.33% (15/180).

The detection rate of neurodevelopmental abnormalities (including neurodevelopmental abnormalities and neurodevelopmental limbic state) in the premature infant group was 26.5%, which was higher than 21.7% in the full-term infant group. The difference was not statistically significant by the chi-square test (*χ*^2^ = 1.155, *P* = 0.283).

An accurate test by Fisher's four-grid table showed that there was no significant difference in the detection rates of CP and hearing injury between the two cohorts (*P* = 0.499). See Table 1 for details.

There was no significant difference in the detection rates of neurodevelopmental abnormalities between the two cohorts by the chi-square test (*χ*^2^ = 1.326, *P* = 0.249). See Table 1.

The detection rate of neurodevelopmental limbic state in the premature cohort was higher than that in the full-term cohort, and the difference was statistically significant by the chi-square test (*χ*^2^ = 6.132, *P* = 0.013), as shown in Table 1.

#### 3.2.2. Comparison of Neurodevelopmental Abnormalities at 12 Months of Age between the Two Cohorts

At the corrected gestational age of 12 months, a cohort of 153 premature infants completed the Gesell test, including 115 cases with normal neurodevelopment and 21 cases with various neurodevelopmental abnormalities, with a detection rate of 13.73%(21/153), including two cases of cerebral palsy (a detection rate of 1.31%, 2/153) and two cases of moderate hearing impairment (a detection rate of 1.31%, 2/153). In the 17 cases with borderline neurodevelopmental state, the detection rate was 11.11% (17/153), as shown in Table 2.

In the 12-month-old full-term cohort, 164 children completed the Gesell test, 142 had normal neurodevelopment, and 9 had language developmental delay (the detection rate was 5.49%, 9/164). In 13 cases with borderline neurodevelopmental state, the detection rate was 7.93% (13/164), as shown in Table 2.

The detection rate of neurodevelopmental abnormalities (including neurodevelopmental abnormalities and neurodevelopmental limbic state) in the premature cohort was higher than that in the full-term cohort, and the difference was statistically significant by the chi-square test (*χ*^2^ = 6.730, *P* = 0.009).

There was no statistically significant difference in the detection rates of CP and hearing impairment between the two cohorts (Fisher's four-grid precision test, *P* = 0.232).

The detection rate of neurodevelopmental abnormalities in the premature infant cohort was higher than that in the full-term infant cohort, and the difference was statistically significant by the chi-square test (*χ*^2^ = 6.269, *P* = 0.012).

There was no significant difference in the detection rates of neurodevelopmental limbic states between the preterm and full-term cohorts (*χ*^2^ = 0.937, *P* = 0.333).

#### 3.2.3. Comparison of Neurodevelopmental Abnormalities between the Two Cohorts at 18 Months of Age

When the gestational age was corrected for 18 months, a cohort of 139 premature infants completed the Gesell evaluation, including 107 cases with normal neurodevelopmental status and 22 cases with various neurodevelopmental abnormalities, with a detection rate of 15.83% (22/139). Among the 10 cases with borderline neurodevelopmental state, the detection rate was 7.19% (10/139). The positive rate of screening in autism spectrum disorder was 7.19% (10/139). See Table 3 for details.

In the 18-month-old full-term cohort, 128 children completed the Gesell evaluation, including 109 cases with normal neurodevelopment and 14 cases with various neurodevelopmental abnormalities, with a detection rate of 10.94% (14/128). There were five cases with borderline neurodevelopmental state, and the detection rate was 3.91% (5/128). The positive rate of autism spectrum disorder screening was 5.47% (7/128). See Table 3 for details.

The difference in the detection rates of neurodevelopmental abnormalities (including neurodevelopmental abnormalities and borderline neurodevelopmental state) between the early birth cohort and the full-term cohort was not statistically significant by the chi-square test (*χ*^2^ = 2.884, *P* = 0.089).

There was no significant difference in the detection rates of neurodevelopmental abnormalities between the premature cohort and the full-term cohort by the chi-square test (*χ*^2^ = 1.366, *P* = 0.243).

There was no significant difference in the detection rates of neurodevelopmental limbic state between the preterm cohort and the full-term cohort by the chi-square test (*χ*^2^ = 1.359, *P* = 0.244).

There was no significant difference in the positive rates of autism spectrum disorder screening between the premature cohort and the full-term cohort by the chi-square test (*χ*^2^ = 0.333, *P* = 0.564).

#### 3.2.4. Comparison of Neurodevelopmental Abnormalities at 24 Months of Age between the Two Cohorts

At the corrected gestational age of 24 months, 172 premature infants in the cohort completed the Gesell test, including 154 cases with normal neurodevelopment and 18 cases with various neurodevelopmental abnormalities, with a detection rate of 10.47% (18/172), including two cases of cerebral palsy (a detection rate of 1.16%, 2/172), two cases of moderate hearing impairment (a detection rate of 1.16%, 2/172), and one case of autism spectrum disorder (a detection rate of 0.58%). See Table 4 for details.

In the 24-month-old full-term cohort, 157 children completed the Gesell evaluation, including 151 cases with normal neurodevelopment and 6 cases with neurodevelopmental abnormalities. All of them were fully developmental delay (language and social backwardness), and the detection rate was 3.82% (6/157). See Table 4 for details.

The detection rate of neurodevelopmental abnormalities in the premature infant cohort was higher than that in the full-term infant cohort, and the difference was statistically significant by the chi-square test (*χ*^2^ = 5.357, *P* = 0.021).

There was no statistically significant difference in the detection rates of CP and hearing impairment between the two cohorts (Fisher's exact four-grid test, *P* = 0.500).

There was no statistically significant difference in the autism spectrum disorder detection rates between the preterm and full-term cohorts (Fisher's four-grid precision test, *P* = 1.000).

### 3.3. Comparison of Development Quotient at the Ages of 6, 12, 18, and 24 Months between the Premature Infant Cohort and the Full-Term Infant Cohort

#### 3.3.1. Comparison of Development Quotient between the Two Cohorts at 6 Months of Age

The scores of adaptive performance area, fine motor energy area, and personal-social energy area in the premature infant cohort at corrected gestational age of 6 months were higher than those in the full-term infant cohort, and the differences were statistically significant upon examination (*P* < 0.05). There was no significant difference in the scores of gross motor energy area and language energy area between the two cohorts (*P* > 0.05), as shown in Table 5.

#### 3.3.2. Comparison of Development Quotient at 12 Months of Age between the Two Cohorts

The scores of adaptive performance area, fine motor energy area, and personal-social energy area in the premature infant cohort at corrected gestational age of 12 months were higher than those in the full-term infant cohort, and the differences were statistically significant upon examination (*P* < 0.05). There was no significant difference in the scores of gross motor energy area and language energy area between the two cohorts (*P* > 0.05), as shown in Table 6.

#### 3.3.3. Comparison of Development Quotient at 18 Months of Age between the Two Cohorts

The scores of adaptive performance area and personal-social energy area in the premature infant cohort at the corrected gestational age of 18 months were higher than those in the full-term infant cohort, and the differences were statistically significant upon examination (*P* < 0.05). There was no significant difference in the scores of gross motor energy area, fine motor energy area, and language energy area between the two cohorts (*P* > 0.05), as shown in Table 7.

#### 3.3.4. Comparison of Development Quotient at 24 Months of Age between the Two Cohorts

The scores of adaptive performance area and personal-social energy area in the premature infant cohort at corrected gestational age of 24 months were higher than those in the full-term infant cohort, and the differences were statistically significant upon examination (*P* < 0.05). There was no significant difference in the scores of gross motor energy area, fine motor energy area, and language energy area between the two cohorts (*P* > 0.05). See Table 8 for details.

## 4. Discussion

### 4.1. Comparison of the Premature Infant Cohort with Full-Term Infant Cohort at Corrected Gestational Ages of 6, 12, 18, and 24 Months

In this study, the developmental quotients of the adaptive performance area, fine motor energy area, and personal-social energy area in the premature infant cohort at the corrected gestational age of 6 months and 12 months were higher than those in the full-term infant cohort, and the differences were statistically significant (*P* < 0.05). There was no significant difference in the scores of large motor energy area and language energy area between the two cohorts (*P* < 0.05). The developmental quotients of adaptive performance area and personal-social energy area at 18 and 24 months of corrected gestational age were higher than those of the full-term infant cohort, and the differences were statistically significant upon examination (*P* < 0.05). There was no significant difference in the scores of gross motor energy area, fine motor energy area, and language energy area between the two cohorts (*P* > 0.05). Yan et al. [10] reported that when the corrected gestational age was 12 months, there was no statistically significant difference in the PDI scores of premature infants with birth gestational ages <32 weeks, 32–33 + 6 weeks, and 34–36 + 6 weeks between each group and the full-term group. Moreover, the MDI scores of the full-term group were lower than those of <32 weeks and 32–33 + 6 groups. At corrected gestational age of 24 months, there were no significant differences in MDI and PDI scores between the preterm of different gestational age groups and the full-term group (*P* > 0.05). Jiang et al. [11] studied the motor and intellectual development trends of premature infants of different birth gestational ages (middle- and late-stage premature infants in the ≥32-week group and early-stage premature infants in the <32-week group) within 24 months of corrected age. The study found that the motor and intellectual development levels of premature infants in the two groups within 24 months of corrected age were significantly lower than that of full-term infants, and both of them could catch up with the full-term infants when correcting 24 months of age. The results of this study were generally consistent with those of the above two studies, namely, the neurodevelopmental levels in the five energy regions of premature infants with gestational age less than 34 weeks and corrected gestational age of 6 months to 2 years after birth were comparable to those of full-term infants The results were consistent with the results of the previous study [12] of our research group and the results of foreign studies [13, 14].

### 4.2. The Detection Rate of Neurodevelopmental Abnormalities at Corrected Gestational Ages of 12 and 24 months in the Premature Infant Cohort Is Higher than That in the Full-Term Infant Cohort

In the 12-month corrected gestational age cohort, there were 153 premature infants, 115 cases with normal neurodevelopment, and 21 cases with various neurodevelopmental abnormalities. The detection rate was 13.73% (21/153), which was higher than 10.47% (18/172) of the full-term cohort (*χ*^2^ = 6.269, *P* = 0.012).

In this study, the detection rate of neurodevelopmental abnormality in the premature infant group at corrected gestational age of 6 months was 26.5%, which was higher than the incidence rate of neurodevelopmental disorder in premature infants of 20.4% reported in the cohort study by Namazzi et al. [15]. This might be related to the fact that the mean gestational age at birth (31.3 weeks) of the premature infant in this study was lower than the mean gestational age at birth (33 weeks) of the premature infant in the study by Namazzi et al. Many studies have shown that the lower the gestational age is, the higher the incidence of neurodevelopmental disorders will be [16, 17].

When the gestational age was corrected for 24 months, there were 172 premature infants in the cohort, 154 cases with normal neurodevelopment, and 18 cases with various neurodevelopmental abnormalities, and the detection rate was 10.47% (18/172), which was higher than that of the full-term infants (3.82%, 6/157), and the difference was statistically significant by Chi-square test (χ2 = 5.357, P = 0.021). The results of this study were consistent with the report by Liang et al. [22].

### 4.3. Pay Attention to the Regular Monitoring of Postnatal Neurodevelopment and Early Education Promotion of Premature Infants with Gestational Age Less than 34 Weeks

The tissues and organs of premature infants are immature and easily damaged by external adverse factors, leading to functional development disorders and abnormalities. Besides, the incidence of premature babies in various countries has an increasing trend, with the incidence rate exceeding 10%. The tissues and organs of premature infants are immature and easily damaged by external adverse factors, leading to functional development disorders and abnormalities. The younger the patient is, the faster the brain develops and the stronger the plasticity will be. The brain has stronger compensation ability for brain injury. It is important to reduce the disability rate and degree of premature infants by adapting early intervention for preterm infants with developmental abnormalities who were born at gestational age less than 34 weeks after birth.

The critical period of brain development is from three months to two years after birth, especially the last three months of the fetus is the most prosperous period of brain development. Premature birth misses the critical period of brain development in the last three months of the fetus. This will cause a reduction in the number of nerve cells, and the pathways of dendritic branching, synapse formation, and cortex thickening are interrupted [18]. This affects the neurodevelopment of premature infants. However, at this stage, the brain has extremely strong plasticity and compensation. Research [19] has shown that giving rich external environment stimulation at this stage can improve the function of the damaged immature brain and the prognosis of premature infants.

To date, the factors contributing to the poor neurological prognosis of premature infants are not fully understood and the results obtained from different studies are different. It is generally believed that the impairment of learning, behavior, and motor ability of premature infants is related to both medical and nonmedical factors [20]. In this cohort study, the premature infants were systematically followed up and the premature infants with abnormal development were given early intervention. The results showed that the detection rate of neurodevelopmental abnormalities in the premature infant group at corrected gestational ages of 12 and 24 months was still higher than that in the full-term infant group. On the other hand, it is related to the fact that the performances of normally developed children in all aspects are parallel, interrelated, and overlapping with each other, while the responses of premature infants are often uneven and significantly different [21]. On the other hand, it is related to the low compliance of parents in the premature infant cohort on early promotion and the insufficient intensity of early education/early promotion in this study, which need to be further studied.

## 5. Conclusion

To sum up, the results of the study showed that the cohort of premature infants with birth gestational age less than 34 weeks had higher adaptive, fine motor, and personal-social energy domain development quotient (DQ) values from the corrected gestational age of 6 months to the corrected gestational age of 24 months after birth, compared with the full-term cohort, and achieved catch-up growth in neurological development, but the detection rate of neurodevelopmental abnormalities at the corrected gestational age of 12 and 24 months was higher than that in the full-term cohort. This study still has many limitations. The detection rate of neurodevelopmental abnormalities in the premature infant group at corrected gestational ages of 12 and 24 months was still higher than that in the full-term infant group. We also need more controlled experiments to explore the reasons for this result. This study only confirms the conclusions of previous studies. We need further research to find the factors contributing to the poor neurological prognosis of premature infants.

Strengthening the systematic management, early promotion and supervision, as well as early intervention for preterm infants with developmental abnormalities who were born at gestational age less than 34 weeks after birth are of great significance to reduce the disability rate and degree of premature infants.

## Figures and Tables

**Table 1:** Comparison of neurodevelopmental outcomes at 6 months of age in a preterm cohort and a full-term cohort.

Cohort	Neurodevelopmental abnormality (*n*)				Neurodevelopmental limbic state (*n*)	Normal neurodevelopment (*n*)	Add up to (*n*)
	Great motor developmental delay	Complete developmental delay	Cerebral palsy break down	Aural comprehension harm			
Premature	9	5	2	2	32	139	189
Mature	6	18	0	0	15	141	180
*X* ^2^	1.326				6.132	1.155	—
*P*	0.249				0.013	0.283	—

**Table 2:** Comparison of neurodevelopment at 12 months between preterm and full-term cohorts.

Cohort	Neurodevelopmental abnormality (*n*)					Neurodevelopmental limbic state (*n*)	Normal neurodevelopment (*n*)	Add up to (*n*)
	Great motor developmental delay	Language retardation	Complete developmental delay	Cerebral palsy break down	Aural comprehension harm			
Premature	2	13	2	2	2	17	115	153
Mature	0	9	0	0	0	13	142	164
*X* ^2^	6.269					0.937	6.730	—
*P*	0.012					0.333	0.009	—

**Table 3:** Comparison of neurodevelopment at 18 months between premature and full-term cohorts.

Cohort	Neurodevelopmental abnormality (*n*)				Neurodevelopmental limbic state (*n*)	Normal neurodevelopment (*n*)	Add up to (*n*)
	Language retardation	Complete developmental delay	Cerebral palsy break down	Aural comprehension harm			
Premature	14	4	2	2	10	107	139
Mature	10	4	0	0	5	109	128
*X* ^2^	1.366				1.359	2.884	—
*P*	0.243				0.244	0.089	—

**Table 4:** Comparison of neurodevelopment at 24 months between preterm and full-term cohorts.

Cohort	Neurodevelopmental abnormality (*n*)				Normal neurodevelopment (*n*)	Add up to (*n*)
	Full development slow	Autism spectrum disorder	Cerebral palsy	Hearing impairment		
Premature	13	One	2	2	154	172
Mature	6	0	0	0	151	157
*X* ^2^	5.357				—	—
*P*	0.021				—	—

**Table 5:** Comparison of neurodevelopmental outcomes between the two cohorts at 6 months of age.

Cohort	Number of cases	Adaptability	Gross motion	Fine motion	Language	Personal-social
Premature	189	92.43 ± 8.54	91.71 ± 10.05	91.25 ± 7.08	96.80 ± 6.40	95.07 ± 8.40
Mature	180	89.96 ± 9.09	91.63 ± 9.47	89.22 ± 9.40	95.88 ± 7.38	90.75 ± 6.03
*T* value		2.694	0.085	2.346	1.283	5.701
*P* value		0.007	0.932	0.020	0.200	0.000

**Table 6:** Comparison of neurodevelopmental outcomes between the two cohorts at 12 months of age.

Cohort	Number of cases	Adaptability	Gross motion	Fine motion	Language	Personal-social
Premature	153	97.26 ± 7.56	95.00 ± 9.44	98.67 ± 7.08	88.10 ± 9.47	96.63 ± 8.64
Mature	164	93.59 ± 3.81	95.62 ± 5.33	94.91 ± 4.05	89.24 ± 7.44	92.26 ± 5.28
*T* value		5.401	−0.708	5.739	−1.179	5.387
*P* value		0.000	0.479	0.000	0.240	0.000

**Table 7:** Comparison of neurodevelopmental outcomes at 18 months of age between the two cohorts.

Cohort	Number of cases	Adaptability	Gross motion	Fine motion	Language	Personal-social
Premature	139	97.82 ± 10.50	97.36 ± 14.27	97.87 ± 10.54	91.53 ± 13.08	98.30 ± 10.64
Mature	128	95.26 ± 6.94	97.27 ± 4.67	97.31 ± 9.71	92.74 ± 12.34	93.14 ± 7.29
*T* value		2.369	0.074	0.449	0.778	4.654
*P* value		0.019	0.941	0.654	0.437	0.000

**Table 8:** Comparison of neurodevelopmental outcomes between the two cohorts at 24 months of age.

Cohort	Number of cases	Adaptability	Gross motion	Fine motion	Language	Personal-social
Premature	172	98.70 ± 4.99	98.34 ± 5.54	99.36 ± 8.334	92.67 ± 9.45	99.24 ± 8.76
Mature	157	96.85 ± 3.41	98.37 ± 3.42	98.44 ± 4.52	92.43 ± 6.06	94.32 ± 4.50
*T* value		3.954	−0.052	1.261	0278	6.494
*P* Value		0.000	0.958	0.208	0.781	0.000

## Data Availability

The data sets used and/or analyzed during the current study are available from the corresponding author on reasonable request.
